# Measuring convergence in the sugarcane industry in China’s Guangxi province

This article has been retracted.

**DOI:** 10.1371/journal.pone.0244617

**Published:** 2021-02-19

**Authors:** Fangfang Zeng

**Affiliations:** 1 Rural Development Institute of Fujian Agriculture and Forestry University, Fuzhou, Fujian, China; 2 Jinshan College of Fujian Agriculture and Forestry University, Fuzhou, Fujian, China; University College London, UNITED KINGDOM

## Abstract

Using the agricultural industry convergence framework, we analyzed the main sugarcane producing areas in China’s Guangxi province from 2010 to 2017. We selected the key elements on sugarcane industry convergence and on the benefit derived from industry convergence and development. We selected six secondary indexes and 18 tertiary indexes and used them to construct an overarching index system for measuring the convergence degree of sugarcane in the primary, secondary, and tertiary industries. We calculated the index’s system weight using the AHP and entropy method, and then the integrated development indicator of the sugarcane industry. Finally, we analyzed the convergence the development stage, achievements, and benefits of the sugarcane industry, as well as the shortage of convergence development. Our findings can provide guidance for the future development of the sugarcane industry in China from the perspective of industry convergence.

## Introduction

In the past decade, agricultural industry convergence has developed rapidly around the world. In large part, agricultural growth has been achieved by promoting the integrated development among the secondary and tertiary agricultural sectors. Existing studies have mainly focused on areas such as connotation, value, mode and path of convergence [1–6]. Xiang-mei Li [7] and Ya-fei Ma [8] evaluated the convergence development of agricultural industry in Beijing, Gansu and other places in China. Fewer studied have focused on the convergence of sugarcane industry. Sugarcane is the main sugar-producing crop in the tropical and subtropical regions of China. The Guangxi province is the most important sugarcane producing area in China. Until 2018, this region was ranked highest in terms of sugarcane yield and harvesting in the entire country. Since 2012, the planting area of sugarcane in Guangxi has been reduced [9]. Owe to the high yield and high sugar content bases construction, sugarcane production capacity grew rapidly. The per unit area yield increased from 6.66 kg/m^2^ in 2011 to 8.14 kg/m^2^ in 2017 [10]. In this paper, we constructed a model to measure the integrated development in the sugarcane industry. We specifically analyzed data of the primary, secondary, and tertiary industry sectors in Guangxi from 2010 to 2017. Based on our results, we made suggestions on how to promote the process of industry convergence in China.

## Research method

### Index system construction

According to existing academic research, promoting industry convergence could expand the agricultural industry chain [11]. In this paper, we constructed an integrated development index for sugarcane industry taking two aspects into consideration: industry convergence achievements and benefits derived from industry convergence [12]. We hope this study would be a useful supplement to the current research. Our index system comprises which consist of the primary, secondary and tertiary index. It is shown in Table 1. Among them, C13 ~ C18 indexes should be explained as follows. Sugarcane industry is the leading agricultural industry in Guangxi, farmers engaged in sugarcane cultivation, processing and sales related industries accounted for up to 70%. The driving benefit of sugarcane industry development is regarded as highly positive correlation with farmers’ income and urban-rural convergence.

**Table 1:** Index table of sugarcane industry convergence.

The Primary Index	The Secondary Index	The Tertiary Index	Index Nature	Calculation Formula
A1 Industry Convergence Achievements	B1Modernization of Sugarcane Planting	C1 Comprehensive Production Capacity of Sugarcane(Kg/m^2^)	Positive	Formula (1)
		C2 Land Productivity(USD/m^2^)	Positive	Formula (2)
		C3 Comprehensive Mechanization Rate of Sugarcane(%)	Positive	Formula (3)
	B2 Ecologization of the Sugarcane Industry	C4 Application Intensity of Pesticide(Kg/m^2^)	Negative	Formula (4)
		C5 Application Intensity of Chemical Fertilizer(Kg/m^2^)	Negative	Formula (5)
		C6 Water Saving Irrigation Coefficient(%)	Positive	Formula (6)
	B3 Sugarcane Industry’s Chain Extension	C7 Ratio of Output Value of Sugar Industry to Output Value of Sugarcane(%)	Positive	Formula (7)
		C8 Profit Margin of Sugar Enterprises(%)	Positive	Formula (8)
		C9 Conversion Rate of Sugarcane in Sugar Industry(%)	Positive	Formula (9)
	B4 Sugarcane Multifunctional Development	C10 Ratio of Output Value of Leisure Agricultural to Output Value of Agricultural (%)	Positive	Formula (10)
		C11 Ratio of Output Value of Sugarcane Productive Service Industry to Output Valueof Sugarcane (%)	Positive	Formula (11)
		C12 Agricultural Credit Input Per Unit (%)	Positive	Formula (12)
A2 Benefits Driven from Industry Convergence	B5 Farmers’ Income	C13 Rural Engel Coefficient(%)	Negative	Formula (13)
		C14 Proportion of Rural Non-agricultural Employment(%)	Positive	Formula (14)
		C15 Cash Income from Sugarcane Production(USD/m^2^)	Positive	Formula (15)
	B6 Urban-rural Convergence	C16 Per Capita Income Ratio of Urban and Rural Areas(%)	Negative	Formula (16)
		C17 Investment Ratio of Fixed Assets Per Capita in Urban and Rural Areas(%)	Positive	Formula (17)
		C18 Rural Financial Expenditure Ratio(%)	Positive	Formula (18)

Sugarcaneyield/sugarcaneplantingarea (1)

Sugarcaneoutputvalue/sugarcaneplantingarea (2)

Machine-ploughinglevel*0.4+machine-broadcastlevel*0.3+machine-harvestinglevel*0.3 (3)

Pesticideconsumptioninsugarcane/sugarcaneplantingarea (4)

Chemicalfertilizerconsumptioninsugarcane/sugarcaneplantingarea (5)

Sugarcanewatersavingirrigationarea/sugarcaneplantingarea (6)

Outputvalueofsugarindustry/outputvalueofsugarcane (7)

Totaloperatingprofit/totalcost (8)

Sugarproduction/rawmaterialquantityofsugarcane (9)

Outputvalueofleisureagricultural/outputcalueofagricultural (10)

Outputvalueofsugarcaneproductiveserviceindustry/outputvalueofsugarcane (11)

Totalagriculturalloans/addedvalueofagriculture (12)

Foodexpenditureofthehousehold/totalconsumptionexpenditureofruralresidents (13)

Ruralnon-agriculturalemployment/ruralnon-agriculturalemployment (14)

Outputvalueofsugarcane-costofsugarcaneproduction (15)

Percapitadisposableincomeofurbanresidents/percapitadisposableincomeofruralresidents (16)

Percapitainvestmentinfixedassetsofruralresidents/percapitainvestmentinfixedassetsofurbanresidents (17)

Ruralfinancialexpenditure/toalfinancialexpenditure (18)

The data used in this study were obtained from the *Statistical Yearbook of Guangxi Zhuang Autonomous Region* (2010–2018), the *Guangxi Yearbook* (2010–2018), and *Compilation of Cost and Income Information of Chinese Agricultural Products* (2010–2018). We used Formula(1) to (18) to deal with the data and calculate the result. It is shown in Table 2.

**Table 2:** Index data of sugarcane industry convergence.

Index / Year	2010	2011	2012	2013	2014	2015	2016	2017
C1	6.66	6.66	6.94	7.20	7.35	7.71	7.85	8.14
C2	0.53	0.53	0.55	0.54	0.46	0.55	0.65	0.68
C3	39.4	41	43.2	46.92	49.82	55	57.11	59.11
C4	11.40*10^−4^	11.55*10^−4^	13.35*10^−4^	16.05*10^−4^	15.30*10^−4^	15.00*10^−4^	14.40*10^−4^	13.95*10^−4^
C5	9.06*10^−2^	8.83*10^−2^	9.34*10^−2^	9.99*10^−2^	9.99*10^−2^	10.28*10^−2^	10.36*10^−2^	9.72*10^−2^
C6	0.12	0.12	0.13	0.13	0.14	0.16	0.17	0.17
C7	0.93	1.13	1.5	1.64	2.05	1.88	1.69	1.88
C8	19.9	21.8	13.6	10.8	10.1	18.2	15.9	18.3
C9	12.06	12.12	12.03	11.78	12.08	12.16	11.51	12.29
C10	0	1.81	3.51	3.59	3.76	3.57	4.14	4.85
C11	27.7	30.36	34.83	37.72	42.56	35.91	31.26	32.02
C12	1.53	1.56	1.82	2.04	2.19	2.26	2.35	2.63
C13	48.50	43.80	42.80	40	36.90	35.40	34.50	32.20
C14	35	36	36	40	34	34	34	35
C15	0.29	0.26	0.23	0.20	0.12	0.21	0.30	0.31
C16	3.76	3.54	3.54	3.43	2.84	2.79	2.73	2.69
C17	10.27	10.54	9.96	9.33	10.2	10.76	30.24	33.69
C18	12.96	12.37	12.36	11.59	11.24	12.24	12.91	13.18

### The evaluation index system

By industry convergence achievements, we refer to the level of agricultural industry upgrading due to the convergence of industries. First, we used the index for the modernization of sugarcane planting to measure the degree to which modern scientific, technological, and managerial practices were applies to agriculture. Second, we used the index for the ecologization of the sugarcane industry to measure the ecological benefits of the industry. Third, we used the index for the sugarcane industry’s chain extension to measure the convergence degree between agriculture and agricultural products processing, sales, and scientific research services. Fourth, we used the index for sugarcane multifunctional development to measure the degree to which diversified choices are provided for improving the industry benefits.

By industry convergence benefits, we refer to the effects of convergence development on the planting areas and on sugarcane growers. First, we used the index for farmers’ income to measure the convergence effect. Second, we used the index for urban-rural convergence to measure the level of social and economic convergence between urban and rural areas.

### Research methods and model construction

There are different kinds of methods available for the comprehensive evaluation of multiple indexes. These could be categorized as subjective and objective methods, each of which has its own advantages and disadvantages. This study adopted a comprehensive weighted evaluation approach, combining the AHP and entropy methods. This approach can overcome the deviation of randomness and conjecture caused by the subjective weighting method. In addition, by using the difference coefficient of the entropy method, the weight value of the subjective weighted evaluation can be modified, this solving the problem of information overlap between multi index variables. Therefore, the weights obtained in this comprehensive way are more scientific [13].

Through consultation with experts, AHP evaluates the importance of an index through pairwise comparison. When the consistency index of the hierarchical total ranking surpasses 0.10, it can be concluded that the results of the hierarchical total ranking are consistent with each other.

The entropy method performs well when it comes to reflecting the variability of index information because it retains the characteristics of index information to the greatest extent. Its calculation formula is shown in Formula (19).

$$e_{j}=-{\left(\text{ln}(m)\right)}^{-1}\sum_{i}^{m}\left(Q_{ij}\times \text{ln}Q_{ij}\right),j=1,2,\cdots ,n$$ (19)

In the formula, m represents the number of evaluated objects, n represents the number of evaluation indexes, *e*_*j*_ represents the entropy of index j, *Q*_*ij*_ represents the proportion of the i-th evaluated object under the j-th index, it is shown in Formula (20).

$$Q_{ij}=x_{ij}/\sum_{i=1}^{m}x_{ij}$$ (20)

On the basis of known entropy, the objective weight of each index could be calculated. Its calculation formula is shown in Formula (21). In the formula, *W*_*j*_ represents the weight of index j.

$$W_{j}=(1-e_{j})/\sum_{j=1}^{n}\left(1-e_{j}\right)$$ (21)

The sugarcane industry convergence is in the dynamic development stage, thus the measurement of its convergence degree needs to be calculated by systematic analysis. The study adopted synthetic indicators method to analyse the convergence development level of sugarcane industry in Guangxi Province. Industry convergence index could be obtained by accumulation. Its calculation formula is shown in Formula (22).

$$ACDIS=P_{1}+P_{2}$$ (22)

In the model, ACDIS represents Agriculture Convergence Development Indicator of Sugarcane, P1 represents indicator of industry convergence achievements, P2 represents indicator of benefits driven by industry convergence. Its calculation formula is shown in Formula (23).

$$P=\sum_{i=1}^{n}\rho_{i}\omega_{i}$$ (23)

In the formula, *P*_*i*_ represents the realization degree of corresponding indicators, *W*_*i*_ represents the weight of each tertiary index. According to different index nature, formula (24) is used to calculate positive index, formula (25) is used to calculate negative index. In the formula, G represents target value, C represents performance value.

$$\rho_{i}=C/G\times 100$$ (24)

$$\rho_{i}=G/C\times 100$$ (25)

### Industry convergence stages

By referring to the relevant literature, such as Yun-Li’s in 2017 and Vieira’s in 2018. The study specifies the division of the sugarcane industry’s convergence stages. It is shown in Table 3.

**Table 3:** Industry convergence stages.

Industry Convergence Stages	Convergence Development Indicators	Industry Convergence Stages	Convergence Development Indicators
Non-integrated Stage	ACDI = 0	-	-
Starting Stage	0≤ACDI<60	Early Stage	0<ACDI≤20
		Middle Stage	20<ACDI≤40
		Later Stage	40<ACDI≤60
Growing Stage	60≤ACDI<80	Early Stage	60<ACDI≤67
		Middle Stage	67<ACDI≤74
		Later Stage	74<ACDI≤80
Initial Convergence Stage	80≤ACDI<100	Early Stage	80<ACDI≤87
		Middle Stage	87<ACDI≤94
		Later Stage	94<ACDI≤100
Deep Convergence Stage	ACDI = 100	-	-

## Results and analysis

### Description of the data

We used the min max normalization method to achieve data standardization. Formula (26) was used to analyze the positive index. Formula (27) was used to is used to analyze the negative index. In the formula, *Y*_*j*_ represents the value of the standardized index, *X*_*j*_ represents the value of the index before standardization, maxX_j_ represents the maximum value in each year for this index, and minX_j_ represents the minimum value in each year for this index. The data processing result is shown in Table 4.

$$Y_{j}=\frac{X_{j}-\text{min}\;X_{j}}{\text{max}\;X_{j}-\text{min}\;X_{j}}$$ (26)

$$Y_{j}=\frac{\text{max}\;X_{j}-X_{j}}{\text{max}\;X_{j}-\text{min}\;X_{j}}$$ (27)

**Table 4:** Standardized value of index data on the sugarcane industry convergence degree.

Index / Year	2010	2011	2012	2013	2014	2015	2016	2017
C1	0.000	0.001	0.191	0.368	0.469	0.708	0.801	1.000
C2	0.311	0.319	0.426	0.379	0.000	0.421	0.881	1.000
C3	0.000	0.081	0.193	0.382	0.529	0.791	0.899	1.000
C4	1.000	0.968	0.581	0.000	0.161	0.226	0.355	0.452
C5	0.850	1.000	0.667	0.240	0.240	0.052	0.000	0.421
C6	0.961	0.950	0.974	1.000	0.964	0.941	0.142	0.000
C7	0.000	0.179	0.509	0.634	1.000	0.848	0.679	0.848
C8	0.838	1.000	0.299	0.060	0.000	0.692	0.496	0.701
C9	0.705	0.782	0.667	0.346	0.731	0.833	0.000	1.000
C10	0.000	0.373	0.724	0.740	0.775	0.736	0.854	1.000
C11	0.000	0.179	0.480	0.674	1.000	0.552	0.240	0.291
C12	0.000	0.027	0.264	0.464	0.600	0.664	0.745	1.000
C13	0.000	0.288	0.350	0.521	0.712	0.804	0.859	1.000
C14	0.167	0.333	0.333	1.000	0.000	0.000	0.000	0.167
C15	0.922	0.764	0.595	0.404	0.000	0.499	0.974	1.000
C16	0.000	0.206	0.206	0.308	0.860	0.907	0.963	1.000
C17	0.039	0.050	0.026	0.000	0.036	0.059	0.858	1.000
C18	0.887	0.582	0.577	0.180	0.000	0.515	0.861	1.000

### Using the minimum relative information entropy method to determine combination weights

After the data standardization, we evaluated the index system using the entropy weighting method. We used the Lagrange multiplier method to optimize the formula for combination weights. Its calculation formula is shown in Formula (28).

$$\bar{W_{j}}={\left(\omega_{j}w_{j}\right)}^{0.5}/\sum_{j=1}^{n}(\omega_{j}w_{j}{)}^{0.5}$$ (28)

In formula(10), $\bar{W_{j}}$ represents the optimize weight value, *ω*_*j*_ represents the weight of AHP, *w*_*j*_ represents the weight of entropy. The result of combination weight is shown in Table 5.

**Table 5:** Weights result for the sugarcane industry convergence evaluation index.

The Primary Index	The Weight of Primary Index(Combination Weight)	The Secondary Index	The Weight of Secondary Index(Combination Weight)	The Tertiary Index	The Weight of Tertiary Index		
					the Weight of AHP	the Weight of Entropy	Combination Weight
Industry Convergence Achievements	0.7758	Modernization of Sugarcane Planting	0.1796	Comprehensive Production Capacity of sugarcane	0.0714	0.053	0.0684
				Sugarcane Land Productivity	0.0714	0.057	0.0709
				Comprehensive Mechanization Rate of Sugarcane	0.0238	0.055	0.0402
		Ecologization of the Sugarcane Industry	0.1103	Application Intensity of Pesticide	0.0156	0.056	0.0329
				Application Intensity of Chemical Fertilize	0.0156	0.054	0.0323
				Water Saving Irrigation Coefficient	0.0311	0.053	0.0451
		Sugarcane Industry’s Chain Extension	0.2942	Ratio of Output Value of Sugar Industry to Output Value of Sugarcane	0.1164	0.051	0.0857
				Profit Margin of Sugar Enterprises	0.0733	0.058	0.0725
				Conversion Rate of Sugarcane in Sugar Industry	0.2771	0.054	0.1360
		Sugarcane Multifunctional Development	0.1918	Ratio of Leisure Agricultural Output Value to Agricultural Output Value	0.1100	0.059	0.0896
				Ratio of Sugarcane Productive Service Industry to Output Valueof Sugarcane	0.0462	0.056	0.0566
				Agricultural Credit Input Per Unit	0.0291	0.058	0.0457
Benefits Driven from Industry Convergence	0.2242	Farmers’ Income	0.1840	Rural Engel Coefficient	0.0164	0.056	0.0337
				Proportion of Rural Non-agricultural Employment	0.0463	0.050	0.0535
				Cash Income from Sugarcane Production	0.0872	0.059	0.0798
		Urban-rural Convergence	0.0402	Per Capita Income Ratio of Urban and Rural Areas	0.0042	0.056	0.0171
				Investment Ratio of Fixed Assets Per Capita in Urban and Rural Areas	0.0026	0.057	0.0135
				Rural Financial Expenditure Ratio	0.0099	0.058	0.0266

### Solution of the convergence index model

To obtain the solution for the convergence index model, we first set the target value as the value specified in the future development plan of the national sugarcane industry. We compared this value with the original index data, and finally obtained the standard value for sugarcane industry convergence. It is shown in Table 6. In order to perceive it intuitively, we used Fig 1 to show the target control value of index data on industry convergence achievements degree. Target control value of index data on benefits driven from industry convergence degree is shown in Fig 2.

**Fig 1:** Target control value of index data on industry convergence achievements degree.

**Fig 2:** Target control value of index data on benefits driven from industry convergence degree.

**Table 6:** Target control value of index data on the sugarcane industry convergence degree.

Index / Year	Target Value	2010	2011	2012	2013	2014	2015	2016	2017
C1	7.5	88.80	88.80	92.53	96.00	98.00	100.00	100.00	100.00
C2	0.92	57.61	57.61	59.78	58.70	50.00	59.78	70.65	73.91
C3	85	46.35	48.24	50.82	55.20	58.61	64.71	67.19	69.54
C4	4.95*10–4	43.42	42.86	37.08	32.35	32.35	33.00	34.38	35.48
C5	3.0*10–2	33.11	33.98	32.12	30.03	30.03	29.18	28.96	30.86
C6	0.56	21.43	21.43	23.21	23.21	25.00	28.57	30.36	30.36
C7	3.0:1	31.00	37.67	50.00	54.67	68.33	62.67	56.33	62.67
C8	30	66.33	72.67	45.33	36.00	33.67	60.67	53.00	61.00
C9	12	100.00	100.00	100.00	98.17	100.00	100.00	95.92	100.00
C10	10	0.00	18.10	35.10	35.90	37.60	35.70	41.40	48.50
C11	20	100.00	100.00	100.00	100.00	100.00	100.00	100.00	100.00
C12	5	30.60	31.20	36.40	40.80	43.80	45.20	47.00	52.60
C13	29.2	60.21	66.67	68.22	73.00	79.13	82.49	84.64	90.68
C14	80	43.75	45.00	45.00	50.00	42.50	42.50	42.50	43.75
C15	0.69	42.03	37.68	33.33	28.99	17.39	30.43	43.48	44.93
C16	1.8	47.87	50.85	50.85	52.48	63.38	64.52	65.93	66.91
C17	25:1	41.08	42.16	39.84	37.32	40.80	43.04	100.00	100.00
C18	9.9	100.00	100.00	100.00	100.00	100.00	100.00	100.00	100.00

According to Formula (22), we calculated the final score, as shown in Fig 3. Both the indicator of sugarcane industry convergence achievements (P1) and the indicator of benefit driven by sugarcane industry convergence(P2) are increasing year by year from 2010 to 2017.

**Fig 3:** Convergence development result for sugarcane.

## Conclusion

### Analyzing of the sugarcane industry convergence stages

As shown in Table 6, the convergence development of the sugarcane industry was in its early stage from 2010 to 2014. In 2015, it was in its growing stage. In large part due to the development of high-quality sugarcane fields, the production capacity of sugarcane in Guangxi has grown rapidly. This indicates that the output value of sugarcane industry in Guangxi has been driven effectively.

### Analyzing the achievements and benefits of the sugarcane industry convergence

As shown in Fig 1, among the tertiary indexes, an indicator score above 80 includes the comprehensive production capacity of sugarcane, the conversion rate of sugarcane in the sugar industry, the ratio of sugarcane productive service industry to output value of sugarcane, and rural financial expenditure ratio. First, our results indicate that the development of high-quality sugarcane fields in Guangxi was successful. Second, by eliminating the backward production capacity of the sugar industry, Guangxi has effectively integrated superior production capacity and laid a foundation the multi-function development. Third, the proportion of sugarcane productive services was far higher than the average level in Guangxi. Thus, these services make a positive contribution in the promotion of promoting sugarcane industry convergence. Fourth, the ratio of rural financial expenditure in Guangxi is higher than the national average level. This indicates that the government could play an important role in promoting the development of the sugarcane industry.

### Analyzing the sugarcane industry convergence restriction factor

As shown in Table 6, among the tertiary indexes, after 2015, an indicator score below 60 includes the application intensity of pesticides, the application intensity of chemical fertilizer, the water saving irrigation coefficient, the ratio of leisure agricultural output value to agricultural output value, the agricultural credit input per unit, the proportion of rural non-agricultural employment, the cash income from sugarcane production, and the investment ratio of fixed assets per capita in urban and rural areas. These factors hinder the comprehensive convergence of the sugarcane industry.

## Suggestions

### Replacing traditional cultivation techniques with modern sugarcane science and technology

China’s sugarcane producing areas are mainly concentrated in the Pearl River Delta, Guangxi, Guangdong, Yunnan, and Hainan [14]. There are several problems with sugarcane production. First, because of poor soil condition, a long period of continuous cropping, and soil degradation, a large amount of fertilizer is applied in order to improve sugarcane yields. Second, due to the small size of the cultivated area, the low educational level of farmers, and the lack of scientific knowledge about fertilization, large amounts of chemical fertilizer are used in an unregulated way. This causes water and land pollution in China [15]. The scope of these problems could be reduced by adopting modern science and technology, reducing the high efficiency cultivation technology, and applying fertilizer in a scientific way. Therefore, we suggest the adoption of modern cultivation technology to replace the traditional sugarcane cultivation method, which involves intensive cultivation and high input with low yield. Under the pressure of mechanization adaption and machine tool selection, sugarcane producers should adopt breeding species and light simplification of production management technology. They should select appropriate sugarcane species to arrange the collocation layout covered during early, middle and late maturing. To improve soil quality, producers should return the filter mud from the sugar factory to the field, as well as the alcohol waste liquor and the broken leaves after the harvest. They should adhere to the implementation of biological control and maintain a healthy ecological environment on their farmland.

The sugarcane industry as a whole needs to adopt modern technology, specifically when it comes to machinery. At present, due to the small area of cultivation and a reduction in the area available for sugarcane production, the mechanical level of the sugarcane industry in China is low. Various management aspects, including field work, ditching, fertilizing, weeding, ridging, and covering, have not yet incorporated technology of high efficiency. Integration in field operation has not been realized due to an incompatibility between agricultural machinery and farm implements. In general, the mechanization level of sugarcane in China is much lower than in Australia, Brazil, the United States, India, Thailand, and South Africa. Due to the poor site conditions and ecological complexity, decision-makers should promote mechanization that is compatible with local conditions through the combination of large and medium sized machinery, as well as by matching agricultural machinery with agronomy.

### Improving the sugarcane industry

Currently, 95% of the sugarcane processing factories in China employ the sulfuric acid method to extract sucrose [16]. The method lags behind more advanced techniques because most sugarcane processing products are bagasse and molasses, so there is a lack of diversity in the by-products. In recent years, the global sugarcane industry has been affected by resource constraints and environmental problems. The most effective way to overcome difficulties and increase competitiveness is to increase the added value of sugarcane by-products and to diversify products. Bagasse is the main by-product of sugarcane, which accounts for about 24 to 27 percent of the total sugarcane product. Using biotechnology for compound enzyme preparation can effectively improve the efficiency of enzymatic hydrolysis for bagasse. In China, Approximately 24 million tons of bagasse are produced annually (equivalent to 14,400,000 tons of dry bagasse). Developing resources for processing bagasse by-products and converting them into high value-added functional materials and biomass chemicals is an effective way to improve the technological level and competitiveness of the sugarcane industry.

### Developing sugarcane-themed tourism services

From the perspective of industrial integration, the development of tertiary industries is an important way to further enhance the comprehensive output value of the sugarcane industry. Sugarcane planting and processing should be combined with leisure tourism [17]. For example, sugarcane could be grown into a variety of labyrinth styles, which visitors could explore and enjoy. Moreover, educational centers could be established where visitors learn about sugarcane growth [18]. At the same time, fruit cane planting should be implemented to provide fresh food. The traditional sugarcane squeezing process should be shown to tourists, allowing them to experience this traditional technique and the satisfaction that comes with squeezing out the sugarcane juice, filtering the bagasse, boiling the sugarcane water, stirring the sugarcane syrup, airing the sucrose, etc. At the same time, producers should utilize modern technology for producing distilled liquor, such as rum, as well as other types of distilled liquor from molasses. The processing mechanism could be displayed and factories can implement tourist sightseeing areas, so that visitors can also see the sugarcane processing mechanism that uses modern technology. Developing a sugarcane culture and encouraging sugarcane planting in suitable areas would help develop sugarcane culture and industry. Decision makers should systematically organize the knowledge on sugarcane planting, the data for its processing technology, as well as traditional folk art materials. These could be stored and displayed in a sugarcane culture exhibition hall, which can serve as a demonstration base for scientific research and education.

### Establishing a more effective mechanism for connecting various participants

Our study revealed that few benefits were derived from the sugarcane industry convergence. While the industrial chain has been extended, a close connection with the industry participants has not been formed. It is necessary for the Chinese government to establish a more effective mechanism for connecting various participants. More consideration should be given to how to connect farmers, cooperatives, and other production organizations as participants in the industrial chain.

## Supporting information

S1 Data (XLS)
